The article "Investigating the Mediating Effect of Patient Self-Efficacy on the Relationship between Patient Safety Engagement and Patient Safety in Healthcare Professionals" was published in 2023. Journal: J Healthc Eng.

# Investigating the Mediating Effect of Patient Self-Efficacy on the Relationship between Patient Safety Engagement and Patient Safety in Healthcare Professionals

**DOI:** 10.1155/2023/8934444

**Published:** 2023-02-21

**Authors:** Xule Wang, Yanli Zhao

**Affiliations:** ^1^Medical College, Xuchang University, No. 1389 Xinghua Road, Xuchang, Henan 461000, China; ^2^Suan Sunandha Rajabhat University, 1 U-Thong nok Road, Dusit, Bangkok 10300, Thailand

## Abstract

Patient safety and involvement of the patients in their safety engagement activities are considered the most important elements in the healthcare professions due to their impact on various individual and organizational outcomes. The study used responses of 456 patients. The simple random sampling (SRS) technique was used to collect data from the respondents. The researcher used individuals as the unit of analysis in this study. The results revealed that patient safety engagement had a positive significant effect on patient safety. When the mediating variable of self-efficacy was analyzed, it showed a significant mediated effect on patient safety. Therefore, it was concluded that self-efficacy mediated the relationship between patient safety engagement and patient safety. The findings of the current study convey that engagement of the patient in the practices for patient safety is predicted through the level of self-efficacy of the patient. The study discussed various implications for theory and practice. The study also discussed potential avenues for future research.

## 1. Introduction

In order to reduce medical mistakes, patient safety and patient participation in safety engagement activities are seen to be the most important aspects [1]. The role of patients to participate and contribute in the error-prevention programs also helps management to effectively manage patient care during hospitalization of the patients. Error-prevention techniques were developed with the purpose of altering how people approach their profession. These methods are meant to be easy to use and, taken together, to emphasize the importance of three fundamental ideas: a personal commitment to safety, close attention to detail, and clear communication. Error reduction includes specific strategies for dealing with complacency, complexity, and the source of mistakes. Recognizing their responsibility, leaders must look for and implement into practice strategies to minimize the chance and consequences of human error. For this, healthcare organizations try to induce patient involvement to improve patient safety [2] as evidenced by the World Health Organization's [3] patient safety campaigns. There are a few studies that have investigated patient involvement to increase patient safety [4]. However, such studies are required to be conducted by scholars to improve patient safety [5]. According to Pursio et al. [5], along with other institutional stakeholders, the patients themselves are required to contribute to their own safety. Therefore, the current study would investigate patients' self-efficacy as a potential mediating factor that mediates the relationship between patient safety engagement activities and patient safety in healthcare organizations. Patient safety depicts the absence of damage, injuries, or harm to the patient which can be carried out through the effective engagement and the involvement of the patient [6]. Since self-efficacy is delineated in a way that it is the process that involves cognition where an individual acquires novel behavioral conducts for the improvement of their capabilities to meet future happening through external environmental and societal influence [7]. So, the desired level of self-efficacy could help to improve the outcomes of the healthcare practice and ultimately the safety of the patient [8]. Davis et al. [9] stated that the elements that assisted to sustain the willingness of the patients to engage in an active manner towards the improvement of the patient safety potentially affected the engagement of patients. According to Davis et al. [9], some important factors of patient safety include the following: (1) patients (personal attributes, knowledge, self-confidence, and self-efficacy), (2) health conditions (nature of the health crisis and severeness of the disease), (3) healthcare workers (the level of their skills, knowledge, and abilities), (4) tasks (patients' safety and patient safety engagement), and (5) workplace setting of healthcare professionals. This study attempted to find out how patient safety engagement and patient safety are interlinked and how patient self-efficacy affects this relationship. Some previous research studies tried to explicate the relationship between patient involvement and patient safety and how to enhance the patient engagement to determine the safety of the patients [4].

The main objective of the study is to analyze the patient's safety engagement and patient safety by means of the patient's self-efficacy. The main aim of the research was to investigate the mediating effect of patients' self-efficacy on the relationship between patient safety engagement and patient safety in healthcare professionals. Therefore, the researcher used quantitative research as the research approach because valid measurement scales are available for the variables of interest in this study.

The paper is organized as follows: Section 2 describes the literature review of the study; the conceptual framework of the study is discussed in Section 3; Section 4 indicates the methodology; Section 5 discusses the data analysis; Section 6 indicates the discussion of the study; and finally, Section 6 describes the conclusion of the study.

## 2. Review of the Literature

### 2.1. Patients' Safety

Aspden et al. [10] defined patients' safety as the act of preventing the inauspicious and unfavorable happening during the provision of healthcare services for the patients. Previous studies described patients' safety as the cognitive procedure or the practice by application of which helps to mitigate the possibilities of unfavorable happening of events that are consequences to the health- or medical-care system [11]. Patient safety is an important aspect of nursing care that aims to reduce preventable mistakes and patient damage. Patient safety is a characteristic of a healthcare system and a group of tried-and-true methods for enhancing treatment. To increase the dependability of care delivery systems, staff can use these safety improvement techniques. However, at present, patients still suffer from accidental injuries or medical damage due to healthcare despite of all medical and technological advancements. At first, it was measured by Brennan et al. [12], and they found that 3.7% of patients were being negatively affected in terms of patient safety. According to Kohn et al. [13], medical and healthcare errors and faults fall between one of the major and greatest reasons for causing serious medical injuries and the death of patients. So, more improvement and advancement in the healthcare sector are deemed necessarily important for the safety of patients as a prime concern. According to Aspden et al. [10], for ensuring the safety of the patients and for the improvement of the healthcare system, the process of reporting of any unusual happening should be stimulated so that lessons could be learned from past errors or faults in order to prevent those same errors in future. Patients' safety can be assured by utilizing and practicing reactive and proactive safety indicators proposed by Reason [14] and improved by Reiman and Pietikäinen [15]. An ongoing need to encourage patient involvement and patient knowledge of patient safety. The study's findings can be used to develop targeted content for educational programs. Prioritizing vulnerable groups within the population will help to increase patient safety and participation [16]. Reactive safety indicators refer to the results, opinions, and judgments drawn and taken out from historic happening of events, for instance, the percentage or the rate at which any certain infection occurs in the patients. On the other hand, proactive safety indicators refer to the close examination and recognition of the factors which could have negative effects on the healthcare organizations in terms of the patients' safety.

### 2.2. Patient Safety Engagement

Patient engagement refers to the act of participation of patients themselves and their families along with the healthcare provider for the amelioration of medical facilities and the healthcare safety [17]. Patient engagement involves encouraging consumers to access educated decisions regarding their own health. Patients who are “activated” or “engaged” exhibit good behavior, such as taking charge of their own health and treatment, and are sometimes referred to as “active patients.” This improves health outcomes while also lowering expenditures. It relieves and facilitates the patient's engagement when the patient is informed about how to maintain their own safety. It is vital to ensure the patient's safety and that they are able to take part in and accept the effort. Willingness and responsiveness relevant to the instructed tasks are needed from the side of patients too [18]. The researchers found that most of the patients are prepared and confident for the engagement in the different sets of activities which are being proposed by the different organizations working for the safety of the patients [19]. The persons who required medical care are uninterrupted observed and monitored by the staff in the hospital but in other circumstances like ambulatory settings, the healthcare provider, family of the patient, and patient himself have the predominant and the opportunities to the greater extent for the promotion of safety in collaboration with the diverse medical care units [20].

According to Hall et al. [21], patients' engagement leads to the betterment and improvement with the help of self-supervision of the medication, creating a design of the patients' reading materials and stuff, and by taking part in the personalized self-management counseling [21]. Due to the patient engagement, novel ideas are being brought by the patients to work in a progressive way [22]. So, this concept of patient engagement be named as a successful widespread drug [23]. As patients present specific and unusual point of view regarding their own health care as being proficient and expert about their own health which assists in the forging of healthcare policies [22]. Patients acknowledged their own health and recognize it in a better way which ultimately leads to better choices related to the healthcare services and the better utilization of the resources [24].

### 2.3. Patient Safety Engagement and Patient Safety

According to the studies of Duhn and Medves [25] and Abid et al. [26], patient safety engagement positively affects patient safety. Therefore, patient safety engagements are encouraged by the scholars and practitioners [25, 26]. In under developing countries, every year around 134 million unfavorable events happening occur due to which 2.6 million people died as a result of unsecured and unsafe medical care [27]. The Development of complications in the procedures and accelerating injuries and damage related to health care give birth to this patient safety discipline. The purpose and intention of patient safety are to mitigate medical risks and to make a reduction in the number of errors and damage to the patients throughout healthcare services while the fundamental principle of this concept is established upon learning from past experiences and inauspicious events [28]. According to the World Health Organization [28], patients' involvement or patients' engagement is one of the prime factors that ascertain the desired outcomes and the successful implementation along with other factors such as the level of skill of healthcare workers, leadership capabilities, and distinct policies and procedures. Lack or absence of confirmation or verification from the side of medical healthcare workers along with the deficiency of patients' involvement and lack of knowledge in patients and lack of patient engagement regarding their own health are the most inherent elements that contribute towards the happening of errors [28]. The following five outcomes are frequently used to evaluate patient safety: errors, adverse events, infections, injuries, and mortality. The final measurements for patient safety that are utilized to describe the harms that patients experience are these results.

Steps taken towards safety engagement in order to ensure the patients' safety depends upon three keen domains: engaging the patients for the detection of the adverse happenings, increasing the confidence of the patients by empowerment for the assurance of the medical care, and accenting the patient engagement as the significant way for the amelioration of the patients' safety [29]. Studies found that the rate of the unfavorable and inauspicious happening can be cut down and patients' safety can be improved with the help of the involvement of the patients and families [26, 29]. In spite of the fact that patients' engagement is the anticipating systematic plan of action for the diminution of errors, it is the merely just transferring and shifting of the irresponsibleness of the safety of the patients from the healthcare provider towards the patients and their family [29].

### 2.4. Patients' Self-Efficacy

Bandura [7] defined self-efficacy as the confidence, sureness, or the feeling of trust of an individual in his or her own abilities and qualities by using which he or she can attain the specific predecided and desired goals and objectives, and this level of confidence regulates the selection, persistency, consistency, and drive of that particular individual towards the accomplishment of the task. Self-efficacy is one of the crucial concepts that help to mediate the practical application of the preacquired knowledge, skills, and abilities for the attainment of desired behavior [30].

Previous studies reflected the self-efficacy of the patients as one of the causal and prime factors for the following medication programs without any interruption [31]. An eminent or higher degree of self-efficacy in the patients leads to higher confidence in them regarding the medication programs and the positive outcomes [32]. Alhalaiqa et al. [33] concluded that the patients possessing a prominent degree of self-efficacy had higher self-confidence and higher chances of rapid recovery. Self-efficacy has been found to be an effective and vital factor that can predict the intent to alter the behavior of the patients [34]. Most individuals are not self-efficacious but their capacity and capabilities to produce the desired effect and results are tied to the specific functioning areas, they have diverse levels of efficacy regarding different functioning areas; an individual who is assured and self-confident in the adoption of the balanced and healthy diet may or may not be assured and confident to that level regarding his capacity for daily exercise, generally, self-efficacy is determined by the circumstances and the requirement of individual [30]. Self-efficacy is the degree to which a person believes in their own skills. Self-efficacy is an excellent indicator of motivation and behavior since it is founded on feelings of control and self-confidence.

### 2.5. Patients' Self-Efficacy as the Mediator of Association between Patients' Safety Engagement and Patients' Safety

Involvement or the engagement of the patient in the practices for patient safety can be predicted through the level of self-efficacy of the patient and capabilities to prevent the flaws and errors related to medical or health care [35]. Most of the scholars stated that the patient engagement is significant for the improvement of the patient safety which ultimately leads to the minimization of the adverse impact of the events on the health of patients, this depends upon the knowledge, information, and medical facts that are known by the patient [36]. The patient engagement framework is the result of nearly 150 professionals in healthcare, human psychology, and technology working together. The framework offers support to healthcare organizations of all sizes and implementation phases. The framework's objective is to assist healthcare organizations in developing care delivery models that are more effective and efficient while placing the needs of the patient first. The patient engagement framework contains five stages, each with its own tools and resources. In regard to engaging patients effectively, the education of healthcare professionals should be assured that they must be clearheaded and free from any type of confusion related to the importance of the role of the patient in patient safety [37]. Previous studies conducted regarding the investigation of the relationship between the patient safety engagement and the patient safety demonstrated that the patient himself/herself and his/her family had distinctive information related to the patient safety of the patient which could yield positive outcomes [38]. Indicators demonstrated that the engagement of the patients facilitated them in the improvement of the patient safety and also assisted in the restraining of the disease [39].

Based upon a critical review of the relevant literature, the researcher framed the following conceptual framework through which hypotheses were also developed.

## 3. Conceptual Framework

To achieve the research objectives, the current study would use the following model (Figure 1):

### 3.1. Hypotheses

On the basis of the conceptual framework, the following hypotheses were developed by the researcher to test them in this study:

**Hypothesis 1 .**

Patient safety engagement directly affects patient self-efficacy.

**Hypothesis 2 .**

Patient self-efficacy directly affects patient safety.

**Hypothesis 3 .**

Patient self-efficacy mediates the relationship between patient safety engagement and patient safety.

## 4. Methodology

The researcher used pragmatism as a research philosophy in the current study due to its applied nature in the current research. Pragmatism is a philosophical movement that comprises individuals who believe that an ideology or concept is true if it functions smoothly, that the significance of a notion may be discovered in the practical implications of recognizing it, and that unrealistic ideas should be avoided. It is characterized as a way of thinking about things that emphasizes a logical or practical solution. Pragmatism, as an example, involves solving issues logically and realistically. The aim of this research was to investigate the mediating effect of patients' self-efficacy on the relationship between patient safety engagement and patient safety in healthcare professionals. Therefore, the researcher used quantitative research as the research approach because valid measurement scales are available for the variables of interest to this study. Those measurement scales would help in getting a quantitative data set which would help the researcher to produce empirical results. Research on health and social care commonly uses quantitative research techniques. They employ objective measures in conjunction with statistical methodologies, mathematics, economic studies, or computational modeling to allow for a systematic, rigorous, empirical examination. Contrarily, qualitative health research involves the gathering and methodical analysis of nonquantitative data regarding people's experiences with health or sickness, and the healthcare system provides a number of strategies that can assist to reduce these risks. The researcher used survey design as an appropriate research strategy because it is directly related to the people who would be involved as the respondent of this study. Moreover, according to Fink [40]; it is better to use survey research as the research strategy when the data is related to the attitudes and behaviors of the people as in the current study the people are involved [41].

The researcher targeted 550 patients admitted to hospitals in China. Among them, only 456 structured self-administered questionnaires were returned that were completely filled-in in all respects. According to Krejcie and Morgan [42], a total of 384 (minimum) sample size was required in this study. Hence, it was considered an appropriate sample size with a confidence interval (alpha) of 5% and a confidence level of 95%. This sample was chosen by using a simple random sampling (SRS) technique to collect data from the respondents. In order to ensure that each sampling unit has an equal probability of being selected, simple random sampling (SRS) selects a sample of *n* sampling units from a population of *N* sampling units. In systematic sampling, all people are chosen at random, as opposed to simple random sampling, which requires that each component of the population be recognized and chosen separately. The researcher used individuals as the unit of analysis. As the researcher used the survey as the research strategy, there was no issue of ethical aspects related to human participants (ethical approval form/consent form) that is necessarily required to be followed in experimental research. The collected data was managed in Statistical Package for Social Sciences (SPSS). For the purposes of group identification, forecasting numerical results, and descriptive statistics, SPSS analyzes data. For effective data management, this tool also features data processing, graphing, and direct marketing features. The main features of SPSS include the ability to create tables and charts with frequency counts or summary statistics over (groups of) cases and variables while using inferential statistics such as ANOVA, regression, and factor analysis. Also, it uses several different file formats for saving data and output. The SPSS files we will utilize in this study fall into three categories: output files (spv), syntax files (sps), and data files (sav). Various tests of descriptive statistics and inferential statistics would be used to find the answers to research questions and to testify the hypotheses. The researcher used measurement scales of self-efficacy (SE) of Elder et al. [43], patient safety engagement of Graffigna et al. [44], and patient safety of Ricci–Cabello et al. [45].

## 5. Data Analysis

### 5.1. Reliability Analysis

The data collected from 456 patients were analyzed with the help of SPSS. Cronbach's alpha measures internal consistency or how closely connected a group of things is. It is regarded as a gauge for the dependability of scales. It is not necessary for the measure to have a “high” value for alpha for it to be one-dimensional. The following reliability statistics (Table 1) are presented to reveal the reliability of the dataset:

SPSS will initially delete all observations with one or more missing values across all variables provided for the current process when a statistical operation is performed. This is referred to as LISTWISE deletion because it is the default procedure. On the basis of the results provided in the tables given above, it was concluded that all the scales had the required level of reliability in the scales used for measuring the variables of interest in this study. Therefore, the researcher went for other analyses.

## 6. Descriptive Statistics

Descriptive statistics are provided in a summary that details the data sample and its measurements and defines, illustrates, and summarizes the key characteristics of a dataset found in the particular research. Reliability analysis may be used to investigate the characteristics of measuring scales and their constituent parts. The reliability analysis approach also generates a number of commonly used scale reliability measures in addition to data on correlations between the scale's individual components. The results of the descriptive statistics of the data (Table 2) collected from the sample of the study are provided in Table 2:

In Table 2, the description of all concerned variables (patient self-efficacy, patient safety engagement, and patient safety) is provided. When the distribution of data values is symmetrical and there are no obvious outliers, it is optimal to utilize the mean. The median should be used when there are obvious outliers or when the distribution of the data values is skewed. The results showed that the means (the average levels) of the variables including patient self-efficacy, patient safety engagement, and patient safety were more than the average level as 4.2789, 4.1075, and 3.7873, respectively. All the mean values were more than the average response. The Valid *N* (listwise) indicates the number of nonmissing values. The variable has *N* valid observations, which is the number of observations. The sum of *N* and the number of missing values equals the total number of observations. These showed that the responses were facing safety issues. However, they had an adequate level of self-efficacy and safety engagement. Moreover, the values of standard deviations and variance were good enough to show minor deviations.

### 6.1. Hypothesis Testing through Mediation Analysis

In order to estimate the effect of independent variables on the dependent variable and to test the hypotheses, the researcher applied mediated regression analysis by running Hay's Macro. Mediation analysis also assumes all of the basic assumptions of the general linear model, such as linearity, normality, error variance homogeneity, and error independence. It is extremely important to double-check these assumptions before doing a mediational study. For significance testing, it either employs the Sobel test or bootstrapping. As this study was aimed at the finding effect, regression analysis was run to test whether or not patient safety engagement significantly affected patient safety and whether patient self-efficacy mediated the relationship between patient safety engagement and patient safety. A proposed causal chain called mediation shows how one variable can impact another, which can then influence a third. The intervening variable, *M*, serves as the mediator. Using regression analysis, a powerful statistical method, you may examine the correlation between two or more important variables. There are many different types of regression analysis, but at its heart, each one examines the impact of one or more independent variables on a dependent variable. The results of the analysis are provided in Table 3:

Results provided in Table 3 show the effect of patient safety engagement (PSE) from the mediating variable self-efficacy (SE). Model fitness is established as the significance value (*p* value) was lower than the threshold value i.e., 0.05. Patient safety engagement (PSE) has a positive effect which is also significant as the significance value (*p* value) was lower than the threshold value i.e., 0.05. Moreover, the *t*-value is also greater than 1.96 i.e., 18.9286. As the values of LLCI and ULCI are not zero and both are positive, it can be inferred that the effect of IV from the mediator is significant.

Results provided in Table 4(the total effect model) show the effect of both the independent variable i.e., patient safety engagement (PSE) and the mediating variable i.e., self-efficacy (SE) on the dependent variable i.e., patient safety (PS). Model fitness is established as the significance value (*p* value) was lower than the threshold value i.e., 0.05. Patient safety engagement (PSE) and self-efficacy (SE) have positive effects which are also significant as the significance value (*p* value) was lower than the threshold value i.e., 0.05 for both the variables. Moreover, the t-values of both the variables are also greater than 1.96 with values of LLCI and ULCI being nonzero and positive. Therefore, it can be inferred that patient safety engagement (PSE) and self-efficacy (SE) have positive effects on patient safety (PS).

Results provided in Table 5 (direct and indirect effects) show the sole effect of patient safety engagement (PSE) on patient safety (PS). Patient safety is a healthcare discipline that developed in response to the increasing complexity of healthcare systems and the associated increase in patient harm in healthcare institutions. In order to provide patients with the best possible treatment, it aims to prevent and minimize risks, mistakes, and injuries. “Patient engagement” is a more comprehensive idea combining patient activation with treatments intended to boost activation and encourage beneficial patient behavior, including the combination of patient activation with treatments intended to boost activation and encourage beneficial patient behavior, including getting regular preventative care or exercise. This effect was significant as the significance value (*p* value) was lesser than the threshold value i.e., 0.05. On the contrary, the indirect or mediated effect of patient safety engagement (PSE) on patient safety (PS) through self-efficacy (SE) as the mediator was significant as shown by the lower limits (BootLLCI) and upper limits (BootULCI) both of them being positive. Therefore, it was concluded that self-efficacy mediated the relationship between patient safety engagement and patient safety. Therefore, all the hypotheses developed by the researcher were accepted by rejecting the null hypotheses of this study.

## 7. Discussions

The current study found significant positive effects of patient safety engagement on the patient safety of the responding patients. This finding is similar to the previous findings of the studies where it was found that patient safety engagement significantly and positively affected patient safety. The studies with similar findings included the WHO [28], Duhn and Medves [25], and Abid et al. [26]. Almost the majority of the studies conducted on this topic found a significant and positive impact on patient safety engagement on patient safety. The current study found that self-efficacy significantly mediated the relationship between patient safety engagement on patient safety. This means that patient safety engagement affected patients' self-efficacy which consequently affected patient safety. Therefore, it was concluded that self-efficacy mediated the relationship between patient safety engagement and patient safety. This finding conveys that the engagement of the patient in the practices for patient safety is predicted through the level of self-efficacy of the patients. This finding is similar to the findings of Lee and Garvin [37], Schwappach [36], Davis et al. [35], Landers et al. [39], and Khan et al. [38].

## 8. Conclusion

The current study recommends healthcare professionals to utilize patient engagement activities in enhancing their safety. The managers, supervisors, and/or organizational leaders can use the findings to guide their contemporary work environments too. The current study also recommends the researcher to lead the research. This study observed various limitations due to limited time and limited financial resources. Those limitations may serve as the opportunities for future research studies. The current study used self-efficacy as the mediating variable that could possibly serve as a booster to enhance patient safety. However, some other variables might also be tested as potential mediators in this relationship such as self-regulation or psychological capital. Additionally, moderating variables may also be tested to clarify the findings of the current study. Future studies may also be conducted by using moderated-mediation or mediated-moderation models while testing and verifying the findings of the current study.

## Figures and Tables

**Figure 1:** Proposed model.

**Table 1:** Cronbach's alpha reliability statistics.

Number of items/questions			Cronbach's alpha
Variables	Patient self-efficacy	5	0.605
	Patient safety engagement	5	0.825
	Patient safety	6	0.674

a. Listwise deletion based on all variables in the procedure.

**Table 2:** Descriptive statistics.

	*N*	Mean		Std. deviation	Variance
	Statistic	Statistic	Std. error	Statistic	Statistic
Patient self-efficacy	456	4.2789	0.01914	0.40880	0.167
Patient safety engagement	456	4.1075	0.02607	0.55671	0.310
Patient safety	456	3.7873	0.02018	0.43103	0.186
Valid N (listwise)	456				

**Table 3:** Mediating effect through self-efficacy.

*Model summary (outcome: SE)*						
*R*	R-Sq	MSE	*F*	Df1	Df2	*p*
0.6641	0.4411	0.0936	358.2901	1.0000	454.0000	≤0.001

*Models*						
	Coeff	Se	*t*	*p*	LLCI	ULCI
Constant	2.2758	0.1068	21.3101	≤0.001	2.0659	2.4856
PSE	0.4877	0.258	19.9286	≤0.001	0.4371	0.5383

**Table 4:** Mediating effect of self-efficacy.

*Model summary (outcome: PS)*						
*R*	R-Sq	MSE	*F*	Df1	Df2	*p*
0.7704	0.5935	0.0758	330.7430	2.0000	453.0000	≤0.001

*Models*						
	Coeff	Se	*t*	*p*	LLCI	ULCI
Constant	0.6418	0.1360	4.7204	≤0.001	0.3746	0.9090
SE	0.3699	0.0422	8.7556	≤0.001	0.2869	0.4529
PSE	0.3805	0.0310	12.2645	≤0.001	0.3195	0.4414

**Table 5:** Direct and indirect effects.

*Direct effect of X on Y*						
	Effect	Se	*t*	*p*	LLCI	ULCI
	0.3805	0.0310	12.2645	≤0.001	0.3195	0.4414

*Indirect effect of X on Y*						
	Effect	Boot se	BootLLCI		BootULCI	
SE	0.1804	0.0198	0.1423		0.2191	

## Data Availability

The data used to support the findings of this study are available from the corresponding author upon request.
